# Using Recursive Feature Selection with Random Forest to Improve Protein Structural Class Prediction for Low-Similarity Sequences

**DOI:** 10.1155/2021/5529389

**Published:** 2021-05-07

**Authors:** Yaoxin Wang, Yingjie Xu, Zhenyu Yang, Xiaoqing Liu, Qi Dai

**Affiliations:** ^1^College of Life Sciences, Zhejiang Sci-Tech University, Hangzhou 310018, China; ^2^Qixin School, Zhejiang Sci-Tech University, Hangzhou 310018, China; ^3^College of Sciences, Hangzhou Dianzi University, Hangzhou 310018, China

## Abstract

Many combinations of protein features are used to improve protein structural class prediction, but the information redundancy is often ignored. In order to select the important features with strong classification ability, we proposed a recursive feature selection with random forest to improve protein structural class prediction. We evaluated the proposed method with four experiments and compared it with the available competing prediction methods. The results indicate that the proposed feature selection method effectively improves the efficiency of protein structural class prediction. Only less than 5% features are used, but the prediction accuracy is improved by 4.6-13.3%. We further compared different protein features and found that the predicted secondary structural features achieve the best performance. This understanding can be used to design more powerful prediction methods for the protein structural class.

## 1. Introduction

Protein structural class is the basic research field in protein research and makes a significant contribution to the research on protein function, protein folding rate, DNA binding site, and protein folding recognition, as well as reducing the search of conformational space and realizing the prediction of the tertiary structure [1–7]. In recent years, the gap between protein sequences and protein structures is becoming larger and larger with the development of sequencing technology, and it is relatively slow to identify three-dimensional structures by experimental methods. Therefore, it is necessary to develop computational methods for fast and accurate determination of protein structural classes.

The protein structures are determined by their sequences. Therefore, protein structure classes can be directly determined based on the sequence information, which can further guide biological experiments and reduce experimental costs. Many protein structural class prediction methods have been proposed since the concept of the protein structure class was put forward [3–5, 7–11]. At first, protein structural class prediction is designed based on the protein composition [1, 12, 13], such as short peptide composition [14–16], pseudo amino acid composition [17–20], and functional domain composition collocation [21]. Amino acid composition (AAC) is calculated according to the ratio of 20 amino acid residues in the sequence and denoted as a numerical vector as the sequence characteristic information [14–16]. However, it did not take the interaction and physicochemical properties of amino acids into account. Pseudo amino acid composition (PseACC) was further proposed as the characteristic information of protein [17–22], which does not merely consider the amino acid residues' composition but also considers the physical and chemical properties such as hydrophobicity of amino acid residues. In addition, the characteristic information is extracted by calculating the peptide components [23], which takes into account the sequence factors among amino acid residues.

The prediction method based on sequence-based features performs well on the high similarity data set, while their precision on the low-similarity data set is only about 50%. Some improved feature extraction methods need to be put forward urgently. Kurgan et al. introduced a SCPRED method with the help of the predicted secondary structures [24]. Zhang et al. calculated a TPM matrix to represent the prediction of secondary structural features [25]. Dai et al. also proposed a statistical feature of the secondary structural features for protein structural class prediction [26]. Ding et al. constructed a multidimensional representing vector as the predicted secondary structure features, and some methods of fuse multiple features are also designed [27]. Chen et al. proposed a multifeature fusion method that combines structural information with physical chemistry [28, 29]. Nanni et al. introduced a prediction method that combines the characteristics of the first-level sequence and the characteristics of the second-level structure [30]. Wang et al. have combined improved simplified PSSM with secondary structural features for protein structural class prediction [31].

With help of the above features, prediction accuracy was improved over 80% for several low-similarity benchmark data sets, but some problems still exist in their development. In order to improve the efficiency of the prediction models, some research integrated different protein features to establish a prediction model. However, it is worth noting that the simple combination of the different features does not necessarily improve the prediction performance. If the combination is not appropriate, it may even offset the information contained in each other, which not only causes the redundancy of information but also increases the complexity and computation of the model.

With the above problems in mind, we proposed a scheme to predict the protein structural classes using the recursive feature selection with random forest. We first explored protein content features, protein position features, reduced combined features, and predicted secondary structural features and discussed their contribution for protein structural class prediction. We then proposed a recursive feature selection method to select important features from the above feature set, where the relative importance index of each feature is calculated based on the random forest algorithm. At last, the features are selected according to their relative importance value. Through a comprehensive comparison and discussion, some novel valuable guidelines for use of the recursive feature selection and protein features are obtained.

## 2. Materials and Methods

### 2.1. Data Sets

Four widely used low-similarity benchmark data sets are selected for comparison with existing methods [24, 25, 32–37]. The first data set is 25PDB, with sequence homology of 25%, which was originally published in [32, 33]. It contains 1673 proteins and domains, which are downloaded from PDB and scanned with high resolution. The second data set is D640, which has 25% sequence identity. It is composed of 640 proteins, and the classification tags are from the SCOP database [32, 33]. The third data set is FC699, in which 858 sequences have 40% low identity. The last data set, denoted as 1189, has 40% sequence identity. It is composed of three-dimensional structure data of 1092 proteins, which are downloaded from the RCSB protein database, and PDB ID is listed in [38].  Table 1 provides more detailed information about these low-similarity benchmark data sets.

### 2.2. Sequence Content Feature

There are a large number of statistical literatures, in which a sequence is interpreted as a series of symbols. A *k*-word is a sequence of *k*-consecutive letters in a sequence. For the sequence *s* with length *m*, the count of *k*-word *w*, represented by *c*(*w*), is the number of times *w* appears in the sequence *s*. Here, the *k*-word is allowed to overlap in the sequence. The sequence content can be described by the frequencies of the *k*-word, and it can be represented by an *n*-dimensional vector C_*k*_^*s*^:

(1) $$\begin{array}{c} {\text{C}}_{k}^{s}=\left(c\left(w_{k,1}\right),c\left(w_{k,2}\right),\cdots ,c\left(w_{k,n}\right)\right), \end{array}$$

where *n* is the total number of all possible *k-*words. Then, the sequence content features can be calculated as

(2) $$\begin{array}{c} {\text{SCF}}_{k}^{s}=\left(\frac{c\left(w_{k,1}\right)}{m-k+1},\frac{c\left(w_{k,2}\right)}{m-k+1},\cdots ,\frac{c\left(w_{k,n}\right)}{m-k+1}\right). \end{array}$$

This work calculates SCF_1_^*s*^ and SCF_2_^*s*^ to construct the sequence content features.

### 2.3. Sequence Position Feature

In addition to the sequence content features, we also pay attention to position distribution of these *k*-word elements. Given a *k*-word, we first transformed a protein structural sequence into several position signal sequences. If the interval distance Dis(*w*_*k*,*i*_) of the given *k*-word *w*_*k*,*i*_ is equal to 1, the consecutive *k*-word *w*_*k*,*i*_ will form a structure and motif domain. Otherwise, they belong to two different domains. Given the Dis(*w*_*k*,*i*_) and the integer *t*, we calculate the probability that Dis(*w*_*k*,*i*_) takes the value *t*, and the probability distribution of the Dis(*w*_*k*,*i*_) will be obtained. The numerical characteristics semimean Semi‐E_*k*_(*w*) and semivariance Semi‐D_*k*_(*w*) are defined by

(3) $$\begin{array}{c} \text{Semi}‐{\text{E}}_{k}\left(w\right)=\overset{t}{\underset{\text{Dis}\left(w_{k}\right)=1}{\sum }}\text{D}\text{is}\left(w_{k}\right)\times \text{P}\left(\text{Dis}\left(w_{k}\right)\right),\\ \text{Semi}‐{\text{D}}_{k}\left(w\right)=\overset{t}{\underset{\text{Dis}\left(w_{k}\right)=1}{\sum }}\left({\left(\text{Dis}\left(w_{k}\right)\right)}^{2}\times \text{P}\left(\text{Dis}\left(w_{k}\right)\right.\right)-{\left[\overset{t}{\underset{\text{Dis}\left(w_{k}\right)=1}{\sum }}\text{D}\text{is}\left(w_{k}\right)\times \text{P}\left(\text{Dis}\left(w_{k}\right)\right)\right]}^{2}. \end{array}$$

The sequence position feature of the standard Semi‐D_*k*_ to Semi‐E_*k*_ is defined as

(4) $$\begin{array}{c} {\text{SPF}}_{k}\left(w\right)=\frac{\text{Semi}‐{\text{E}}_{k}\left(w\right)}{\text{Semi}‐{\text{D}}_{k}\left(w\right)}. \end{array}$$

SPF_*k*_(*w*) is the variability of the *k*-word *w* in relation to its population mean [26], and we calculate SPF_1_(*w*) and SPF_2_(*w*) to construct the sequence position features.

### 2.4. Reduced Sequence Feature

Hydrophilicity is an important physical and chemical property of amino acids. According to the hydrophilicity of amino acids, 20 kinds of amino acids can be divided into three categories: internal group, external group, and ambivalent group. The reduction of protein sequences is defined according to the following rule:

(5) $$\begin{array}{c} F\left(S\left(i\right)\right)=\left\{\begin{array}{cc} I, & \text{if }S\left(i\right)=F,I,L,M,V,\\ E, & \text{if }S\left(i\right)=D,E,H,K,N,Q,R,\\ A, & \text{if }S\left(i\right)=D,E,H,K,N,Q,R, \end{array}\right. \end{array}$$

where *S*(*i*) represents the *i*-th letter in protein sequence *s* and *F*(*S*(*i*)) represents the substitution for *S*(*i*).

With help of the *F*(*S*(*i*)), a protein sequence can be transformed into a reduced sequence, which contains only three letters I, E, and A. For example, given a protein sequence *S* = *ESHFTCISLNEYAMQ*, we can get its reduced protein sequence *F*(*S*) = *EAEIAAIAIEEAAIE*. Here, we calculate the sequence composition and position features of the reduced sequence to combine reduced sequence features.

### 2.5. Predicted Secondary Structural Features

The protein sequence feature achieves promising results in the protein structural class prediction, but its accuracy is limited. Some studies have shown that the content and spatial arrangement of secondary structural elements are also important factors affecting the complex function or structure of proteins. Therefore, one of the methods to improve the prediction accuracy is to add secondary structural features to the feature set [24–31]. In this work, PSI-PRED is used to predict the secondary structure sequence [39], and the 11 widely used predicted secondary structural features are calculated to improve protein structural class prediction [40].

1. Predicted secondary structure element content (content_SE_): given a predicted secondary structure, the content of its predicted secondary structure elements content_SE_ can be calculated by the following formula

(6) $$\begin{array}{c} {\text{content}}_{\text{SE}}=\frac{{\text{Count}}_{\text{SE}}}{\sum_{x\epsilon \left\{C,H,E\right\}}{\text{Count}}_{x}}. \end{array}$$

*H*, *E*, and *C* denote *α*-helix, *β*-strand, and coil, respectively.

(2) First- and second-order composition moment vector (CMV), another important structure feature, can be calculated as follows:

(7) $$\begin{array}{c} {\text{CMV}}_{\text{SE}}^{k}=\frac{\sum_{j=1}^{{\text{Count}}_{\text{SE}}}{\text{PO}}_{{\text{SE}}_{j}}^{k}}{\prod_{d=1}^{k}\left(N-d\right)}, \end{array}$$

where PO_SE_*j*__^*k*^ denotes the secondary structure element at the *j*-th position in the secondary structure sequence with length *N*, and *k* is the vector order.

(3) Length of the longest segment (MaxSeg_SE_):

(8) $$\begin{array}{c} {\text{MaxSeg}}_{\text{SE}}=\text{MaxLen}\left(\text{SEG}:{\text{SEG}}_{\text{SE}}\right), \end{array}$$

where MaxLen denotes the maximal segment length function and SEG_SE_ is the segments that consist of the structure element SE.

(4) Normalized length of the longest segment (NMaxSeg_SE_):

(9) $$\begin{array}{c} {\text{NMaxSeg}}_{\text{SE}}=\frac{\text{MaxLen}\left(\text{SEG}:{\text{SEG}}_{\text{SE}}\right)}{N}, \end{array}$$

where *N* is the sequence length.

(5) Average length of the segment (AvgSeg_SE_):

(10) $$\begin{array}{c} {\text{AvgSeg}}_{\text{SE}}=\frac{\sum \text{L}\text{en}\left(\text{SEG}:{\text{SEG}}_{\text{SE}}\right)}{{\text{Content}}_{{\text{SEG}}_{\text{SE}}}}, \end{array}$$

where Len is the segment length function and Content_SEG_SE__ denotes the content of the SEG_SE_.

(6) Normalized average length of the segment (NAvgSeg_SE_):

(11) $$\begin{array}{c} {\text{NAvgSeg}}_{\text{SE}}=\frac{\sum \text{L}\text{en}\left(\text{SEG}:{\text{SEG}}_{\text{SE}}\right)}{N\times \text{Conten}{\text{t}}_{{\text{SEG}}_{\text{SE}}}}, \end{array}$$

where *N* is the sequence length.

(7) Alternating frequency of *α*-helices and *β*-strands and proportion of parallel *β*-sheets and antiparallel  *β*-sheets (APPA).

Liu and Jia compared the alternating frequencies of different structure elements and found that the *α*-helices and *β*-strands alternate more frequently in *α*/*β* proteins than in *α* + *β* proteins, so they introduced the alternating frequency of the *α*-helices and *β*-strands to predict protein structural class [35]. The normalized alternating frequency is defined as follows:

(12) $$\begin{array}{c} {\text{NAlt}}_{\text{SE}}=\frac{{\text{Content}}_{\alpha -\beta }}{\text{SeqLen}}, \end{array}$$

where Content_*α*−*β*_ denotes the total alternation of the  *α*-helices and *β*-strands, and SeqLen is the sequence length.

### 2.6. Recursive Feature Selection with Random Forest

Each decision tree in the random forest is divided into training sets from the root node according to the top-down principle. The root node of the tree is divided into left and right nodes according to the principle of maximum information gain, that is, the training data of the node is divided into two subsets. Under the same rule, the remaining nodes continue to split until the branch stop rule is satisfied. Among them, node information gain can be calculated by information entropy, information gain rate, and Gini index. In this study, information entropy is selected to obtain information gain, which is defined as follows:

(13) $$\begin{array}{c} \text{IG}\left(S,A\right)=\text{Entropy}\left(S\right)-\text{Entropy}\left(S,A\right), \end{array}$$

where

(14) $$\begin{array}{c} \text{Entropy}\left(S\right)=-\overset{c}{\underset{i=1}{\sum }}p\left(i\right)\log_{2}\left(p\left(i\right)\right),\\ \text{Entropy}\left(\text{S},\text{A}\right)=\underset{v\in \text{values}\left(A\right)}{\sum }\frac{\left|S_{v}\right|}{\left|S\right|}\text{Entropy}\left(S_{v}\right), \end{array}$$

where *S* is the training set with the number of categories *c*, *A* is the characteristic attribute, *p*(*i*) is the probability of the class *i* in *S*, *i* = 1, ⋯, *c*. *S*_*v*_ is the *S* subset of attribute *A*, |*S*_*v*_| is the number of statistical samples, and |*S*| is the number of samples of training set *S*. In this study, there are four types of problems; thus, *c* = 4.

For the decision tree classifier, the classification rate is an important index to measure the constructed classifier, but the importance of feature information in the construction of the decision tree node cannot be ignored. In order to select the important features with a strong classification ability, this work introduces the idea of random forest feature selection based on relative importance.

In the experiment, a certain number of features are randomly selected from the candidate features to construct a large number of decision trees, so as to select representative and effective feature information. Firstly, the *d* candidate features obtained from different feature extraction methods are randomly divided into *s* subsets. In each subset, 50% of the samples corresponding to *m* features are randomly selected as the training sample subset, and the remaining 50% as the test sample subset, which are, respectively, used to construct the classification tree and evaluate the performance of the classification tree, *t* times in total. After the above two steps, a total of *st* decision trees are generated, in which *s* and *t* must be large enough, especially *s*. Each feature information has a chance to appear in different subsets, and it also makes the selected feature information more accurate.

In order to measure the relative importance of the extracted features, the weighted classification rate is used to evaluate the classification ability of the decision tree on the test set. For a class *c* classification problem, let *n*_*ij*_ be the number of class *i* samples divided into class *j* samples, *i*, *j* = 1, ⋯, *c*. In this way, the weighted classification rate introduces the size of each class sample set. The specific definition is as follows:

(15) $$\begin{array}{c} w=\frac{1}{c}\overset{c}{\underset{i=1}{\sum }}\frac{n_{ii}}{n_{i1}+n_{i2}+\cdots +n_{ic}}. \end{array}$$

In the decision tree, if a feature contains more information, it will play a greater role in the classification rate of the decision tree and gain more information. Therefore, the relative importance (RI) index of a feature is defined as

(16) $$\begin{array}{c} {\text{RI}}_{g_{k}}=\overset{st}{\underset{\tau =1}{\sum }}w\underset{n_{g_{k}}}{\sum }\text{I}\text{G}\left(n_{g_{k}}\left(\tau \right)\right)\left(\frac{\text{no}.\text{in}{\text{n}}_{g_{k}}\left(\tau \right)}{\text{no}.\text{in}\tau }\right), \end{array}$$

where *w* is the weighted classification rate of a decision tree. In the *st* decision trees of random forest, *g*_*k*_ is the relatively important feature generated in the *τ* tree. All nodes are denoted as *n*_*g*_*k*__(*τ*), IG(*n*_*g*_*k*__(*τ*)) and no.inn_*g*_*k*__(*τ*) are labeled as the information gain and sample number of the nodes, and no.in*τ* is the number of roots of the *τ* tree. The RI value of each feature is calculated using the above method, and then, the features are sorted according to the RI value. Finally, the representative feature information with great contribution can be selected.

### 2.7. Classification Algorithm

Support vector machine (SVM) is a large edge classifier based on statistical learning theory. It uses an optimal separation hyperplane to separate two kinds of data. For the binary support vector machine, the decision function is

(17) $$\begin{array}{c} f\left(x\right)=\overset{N}{\underset{i=1}{\sum }}\alpha_{i}y_{i}K\left(x_{i},x\right)+b, \end{array}$$

where *b* is a constant, *C* is a cost parameter controlling the trade-off between allowing training errors and forcing rigid margins, y_*i*_*ϵ*{−1, +1}, *x*_*i*_ is the support vector, 0 ≤ *α*_*i*_ ≤ *C*, and *K*(*x*_*i*_, *x*) is the kernel function. This paper uses Vapnik's support vector machine to predict protein structural classes [41]. Since protein has more than two structural classes, we choose the “one-to-one” strategy of multiclass SVM. Given an unknown class of test protein, we calculate the combined features and select the efficient features based on the recursive feature selection with random forest. The support vector machine will then find an optimized linear partition to solve this multiclass problem.

This work chooses the Gauss kernel function of the support vector machine because of its superiority in solving nonlinear problems [42, 43]. Furthermore, a simple grid search strategy is used to select the parameters *C* and gamma with the highest overall prediction. It is designed based on 10 times cross-validation of each data set, and the values of *C* and gamma are taken from the 2^−10^ to 2^10^.

### 2.8. Performance Evaluation

There are three widely used cross-validation methods (subsampling test, independent data set test, and jackknife test) to evaluate the classifier's ability. The jackknife test always produces a unique result, which helps to check the quality of various prediction methods. Therefore, we chose the jackknife test to evaluate the proposed method and introduced the sensitivity (Sens), specificity (Spec), and F1 as standard performance indicators, as well as the accuracy and overall accuracy of each category. These standard performance indicators are defined as follows:

(18) $$\begin{array}{c} {\text{Accuracy}}_{i}=\frac{{\text{TP}}_{i}}{\;|\;C_{i}\;|\;},\\ \text{Overall accuracy}=\frac{\sum {\text{TP}}_{i}}{\sum \;|\;C_{i}\;|\;},\\ \text{Sens}=\frac{\text{TP}}{\text{TP}+\text{FN}},\\ \text{Spec}=\frac{\text{TN}}{\text{FP}+\text{TN}},\\ \text{F}1=\frac{2\text{TP}}{2\text{TP}+\text{FN}+\text{FP}}, \end{array}$$

where TP is the number of true positives, FP is the number of false positives, TN is the number of true negatives, FN is the number of false negatives, and ∣*C*_*i*_∣ is the number of proteins in each structural class *C*_*i*_ (all-*α*, all-*β*, *α*/*β* and *α* + *β* classes).

## 3. Results and Discussion

### 3.1. Performance of Proposed Prediction Method

The low sequence homology of 25PDB, D640, FC699, and 1189 was 25%, 25%, 40%, and 40%, respectively. A simple grid search strategy is adopted for *C* and gamma values based on the 10 times cross-validation of each data set. The sensitivity (Sens), specificity (Spec), and F1 of the proposed method are summarized in Table 2.

Table 2 shows that the prediction performance of the all-*α* class is the best among the four structural classes, and its sensitivity, specificity, and F1 are higher than 90%. But the lower predictions are related the  *α* + *β* class. From Table 3, we find that the overall accuracy of the method is more than 86% for the four data sets. The overall accuracy of the all-*α* class was significantly higher than that of other categories, and the accuracy was more than 94%, followed by all categories and categories. It is not difficult to find that the average total accuracy of the *α* + *β* class of the four data sets is 86.1%, which is 10% lower than that of all classes. These results indicate that it is more difficult to predict the *α* + *β* class because of the nonnegligible overlap in this category.

### 3.2. Performance Comparison with the Competing Predictions

This paper further compared the proposed method with the available competing methods. Here, the accuracy of each class and the overall accuracy are chosen as evaluation indexes to evaluate all the prediction methods, and their results are summarized in Table 3. The proposed method is first compared with AADP-PSSM [44], AAC-PSSM-AC [45], and Ding et al.'s method [46] based on the position-specific scoring matrix. Among all the experiments, the proposed method achieves the best performance, with accuracy above 5.4-12.5% better than the next competing Ding et al.'s method [46].

As for the 25PDB data set, we further compare the proposed method with the competitive methods: SCPRED [32, 33], MODAS [34], S. Zhang et al. [25], RKS-PPSC [47], Ding et al. [48], Xia et al. [49], L.C. Zhang et al. [36], and S.L. Zhang et al. [16]. It is easy to note that the proposed method achieves the best performance, and the overall accuracy is 91.5%, which is 7.2 percentage points higher than Ding et al.'s method [48]. In D640 data sets, we compare the proposed method with SCEC [38], SCPRED [32, 33], RKS-PPSC [47], Zhang et al. [16], and Kong et al. [20]. The overall accuracy of our method is 91.7%, which is 7-8.1% higher than other competitive methods [16, 20]. As for FC699, the comparison is performed between the proposed method and SCPRED [32, 33], 11 features [35], and Kong et al. [20]. We find that the overall accuracy of this method is 96.7%, which is significantly better than other methods. In the 1189 experiment, SCPRED [32, 33], MODAS [34], RKS-PPSC [47], L.C. Zhang et al. [36], S.L. Zhang et al. [16], and Kong et al. [20] are compared with the proposed method, and we find that the proposed method achieves the best performance among all the competing methods. It is the only prediction method with an overall accuracy of more than 86%, which is 3.1% higher than other competitive methods.

It can be seen from Table 3 that the prediction accuracy of *α*/*β* class has been improved. Specifically, the accuracies of the *α* + *β* class for 25PDB, 1189, 640, and FC699 data sets are 85.7%, 80.7%, 96.3%, and 81.7%, respectively, which are 10.2%, 3.5%, 12.1%, and 8.3% higher than those of the next competitive method, respectively [16, 20]. These results show that the proposed method outperforms the available PSSM-based and PSSM-free prediction methods, indicating that the recursive feature selection with the random forest can select important features from the combined feature set and advances predict precision. This understanding can be used to develop more powerful protein structure prediction methods.

### 3.3. Influence of Recursive Feature Selection

A feature of the proposed method is the recursive feature selection with random forest, which calculates the RI value of each feature and selects the representative features with great contribution. For a better understanding of the recursive feature selection, we select the feature set with size from 10 to 857. All experiments are performed with each selected feature set using the jackknife cross-validation test, and the overall accuracy is chosen to represent the score in this prediction.  Figure 1 shows the overall accuracies of all experiments with the selected feature sets for four data sets.

As would be expected, the overall accuracy first increases and then decreases as the selected feature size continues to increase. When the selected feature set size is less than 50, all data sets have reached the best prediction. As the number of selected features increases, the overall accuracy will decrease. The number of selected features corresponding to the best performance is far less than the total number of original features. Therefore, there is a large amount of redundant information in the original combination feature set. After the recursive feature selection with the random forest is used to select and reduce the dimension, the classification rates of four data sets 25PDB, 1189, 640, and FC699 are 91.5%, 86.6%, 91.7%, and 96.7%, respectively, which increased by 4.6-13.3%.

### 3.4. Influence of the Different Features

To improve the prediction of protein structural classes, we use four kinds of protein features: protein sequence features, protein position features, reduced combined features, and predicted secondary structure features. For brevity, let PSF, PPF, RCF, and PSSF denote these four kinds of protein features, respectively. Through the experiments, we want to address which features contribute to the prediction better.

To evaluate the contribution of each kind of the protein features, we present the comparison of the overall prediction accuracies of four kinds of the protein features in Figure 2. It indicates that each feature makes its own positive contributions to the predictions. PSSF achieves the best performance among the four kinds of the protein features, which is 8%~31% higher than the other three features. In addition, PSSF are selected as the efficient features, which indicates that PSSF is relatively important and has a great contribution to the improvement of prediction. It is easy to note that PSSF is directly extracted from the predicted secondary structure sequences, including the information of *α*-helix and *β*-fold alternation frequency and spatial arrangement. Compared with the amino acid frequency and position, the secondary structure sequence information is more closely related to the secondary structure types; this is why it achieves the best performance in protein structure prediction.

## 4. Conclusion

Protein structural classes provide some useful information for the study of the whole folding type, especially for proteins with low sequence similarity. Various types of protein features are combined to improve the protein structural class prediction. However, it should be noted that the feature fusion will also bring information redundancy and affect the efficiency and accuracy of prediction. This paper proposed a feature selection method for protein structural class prediction, which calculates the RI value of each feature with the random forest and selects the representative features based on each contribution. To do so, we first extracted protein sequence features and protein position features, reduced combined features, predicted secondary structure features, and used the recursive feature selection with random forest to select the core features for prediction. The experiment results show that the recursive feature selection with the random forest effectively improves the efficiency of protein structural class prediction. Only less than 5% features are used, but the prediction accuracy is improved by 4.6-13.3%. For a better understanding of different protein features, we compared the contribution of each kind of the protein features and found that the predicted secondary structural features achieve the best performance among the four kinds of the protein features, which is 8%~31% higher than the other features. This understanding can be then used to develop more powerful methods for protein structural class prediction.

## Figures and Tables

**Figure 1:** The comparison of the overall accuracies of all experiments with the selected feature sets for four data sets.

**Figure 2:** Comparison of the overall prediction accuracies of four kinds of the protein features.

**Table 1:** Protein distribution of different structural classes among four protein data sets.

Data set	All-*α*	All-*β*	*α*/*β*	*α* + *β*	Total
25PDB	443	443	346	441	1673
D640	138	154	177	171	640
FC699	130	269	377	82	858
1189	223	294	334	241	1092

**Table 2:** Sensitivity (Sens), specificity (Spec), and F1 of the proposed method on four data sets.

Data set	Class	Sens (%)	Spec (%)	F1 (%)
25PDB	All-*α*	94.81	98.29	95.02
	All-*β*	95.26	98.13	95.05
	*α*/*β*	89.88	95.25	86.39
	*α* + *β*	85.71	97.16	88.52
D640	All-*α*	97.10	97.81	94.70
	All-*β*	92.86	99.18	95.02
	*α*/*β*	97.18	92.87	90.05
	*α* + *β*	80.70	98.93	87.90
FC699	All-*α*	97.69	99.45	97.32
	All-*β*	98.51	99.49	98.70
	*α*/*β*	95.23	99.38	97.16
	*α* + *β*	96.34	97.68	88.27
1189	All-*α*	94.62	96.55	90.95
	All-*β*	89.80	98.50	92.63
	*α*/*β*	82.04	94.20	84.05
	*α* + *β*	81.74	92.95	79.12

**Table 3:** Prediction accuracies (variances in the brackets) of the proposed method for four data sets and comparison with other reported results.

Data set	Method	Prediction accuracy (%)				
		All-*α*	All-*β*	*α*/*β*	*α* + *β*	Overall
25PDB	AADP-PSSM [44]	69.1	83.7	85.6	35.7	70.7
	AAC-PSSM-AC [45]	85.3	81.7	73.7	55.3	74.1
	SCPRED [32, 33]	92.6	80.1	74.0	71.0	79.7
	MODAS [34]	92.3	83.7	81.2	68.3	81.4
	RKS-PPSC [47]	92.8	83.3	85.8	70.1	82.9
	Ding et al. [46]	95.0	81.3	83.2	77.6	84.3
	Xia et al. [49]	92.6	72.5	71.7	71.0	77.2
	Zhang et al. [36]	95.7	80.8	82.4	75.5	83.7
	Ding et al. [48]	91.7	80.8	79.8	64.0	79.0
	Zhang et al. [16]	94.4	83.3	83.5	73.2	83.6
	This paper	94.8	95.3	89.9	85.7	91.5
D640	SCEC [38]	73.9	61.0	81.9	33.9	62.3
	SCPRED [32, 33]	90.6	81.8	85.9	66.7	80.8
	RKS-PPSC [47]	89.1	85.1	88.1	71.4	83.1
	Ding et al. [46]	92.8	88.3	85.9	66.1	82.7
	Zhang et al. [16]	92.0	81.8	87.6	74.3	83.6
	Kong et al. [20]	94.2	80.5	87.6	77.2	84.5
	This paper	97.1	92.8	97.1	80.7	91.7
FC699	SCPRED [32, 33]	—	—	—	—	87.5
	11 features [35]	97.7	88.0	89.1	84.2	89.6
	Kong et al. [20]	96.2	90.7	96.3	69.5	92.0
	This paper	97.7	98.5	95.2	96.3	96.7
1189	AADP-PSSM [44]	69.1	83.7	85.6	35.7	70.7
	AAC-PSSM-AC [45]	80.7	86.4	81.4	45.2	74.6
	SCPRED [32, 33]	89.1	86.7	89.6	53.8	80.6
	MODAS [34]	92.3	87.1	87.9	65.4	83.5
	RKS-PPSC [47]	89.2	86.7	82.6	65.6	81.3
	Zhang et al. [36]	92.4	84.4	84.4	73.4	83.6
	Ding et al. [46]	89.2	88.8	85.6	58.5	81.2
	Zhang et al. [16]	91.5	86.7	82.0	66.4	81.8
	Kong et al. [20]	91.9	84.4	85.3	72.2	83.5
	This paper	94.6	89.7	82.1	81.7	86.6

## Data Availability

All the data used to support the findings of this study are available on https://github.com/qidaizstu/recursive-feature-selection.
